# Meta-Analysis of Naoxintong Capsule for Patients with Vascular Dementia

**DOI:** 10.1155/2022/5000948

**Published:** 2022-07-06

**Authors:** Li Li, Yawei Zheng, Jinjing Bao, Yandong Zhao, Qiuchi Zhang, Wenlei Li, Minghua Wu

**Affiliations:** ^1^Jiangsu Province Hospital of Chinese Medicine, Nanjing, China; ^2^Affiliated Hospital of Nanjing University of Chinese Medicine, Nanjing, China; ^3^Nanjing University of Chinese Medicine, Nanjing, China

## Abstract

**Background:**

Vascular dementia (VaD) is the second most common form of dementia among the elderly. There is currently no unequivocal recommendation of an effective treatment option for VaD.

**Objective:**

The purpose of this study was to evaluate the efficacy and safety of Naoxintong capsule (NXT) in the treatment of VaD patients.

**Methods:**

We searched for randomized controlled trials (RCTs) published before September 2021 in PubMed, Embase, Web of Science, Cochrane Library, CNKI, VIP, and Wanfang databases. The trials assessed the efficacy and/or safety of NXT in treating patients with VaD. A meta-analysis was then performed using Stata 14.0 software.

**Results:**

A total of 33 studies comprising 2,947 patients with VaD were included in this study. The meta-analysis revealed that NXT improved cognitive function in VaD patients, increased the mini-mental state examination (MMSE) score by 3.33 points (WMD = 3.33, 95% CI (2.72, 3.94)), the Montreal Cognitive Assessment (MoCA) score by 4.31 points (WMD = 4.31, 95% CI (2.72, 5.90)), and the Hasegawa dementia scale (HDS) by 2.71 points (WMD = 2.71, 95% CI (1.26, 4.17)). Furthermore, NXT significantly improved the daily lives of VaD patients, lowering the activities of daily living (ADL) score by 5.85 points (WMD = −5.85, 95% CI (−7.03, −4.66)). NXT improved the total effective rate (TER) (OR = 2.62, 95% CI (2.09, 3.29)) of the patients without increasing the occurrence of adverse events (AEs; OR = 0.72, 95% CI (0.43, 1.22)). Subgroup analysis revealed that whether NXT was used alone or in combination with western medicine, it could enhance the overall curative effect.

**Conclusions:**

NXT may be an effective and safe treatment option for VaD. However, because of the limited number and quality of articles included, this study's findings need to be validated by additional high-quality, large-sample, and multicenter RCTs (Systematic Review Registration Number: PROSPERO; https://clinicaltrials.gov/ct2/show/CRD42021233199).

## 1. Introduction

Vascular dementia (VaD) is a condition characterized by clinical or subclinical cerebrovascular damage induced by an ischemic/hemorrhagic stroke or other cerebrovascular diseases. VaD is the second most common cause of dementia in the elderly [1]. The prevalence of VaD increases with age, and the risk doubles after every five years [2]. Cerebrovascular disease and associated risk factors (hyperlipidemia, hypertension, diabetes, or smoking), as well as ischemic white matter disease, are factors that fuel the development of VaD [3, 4]. The primary pathological mechanism for VaD is decreased cerebral blood perfusion [5]. Cerebral ischemia and hypoxia can cause brain tissue loss, resulting in cognitive and memory impairment [6]. Apart from memory loss, VaD causes language deficits and impaired executive functions or emotional changes, impairing families' and society's capacity to operate daily [7].

Currently, there is no treatment guideline approved by the Food and Drug Administration (FDA) for the treatment of VaD [8]. The available treatment options for VaD are aimed at addressing the modifiable VaD risk factors such as hypertension, diabetes, smoking, and atherosclerosis or at delaying disease progression and alleviating behavioral symptoms such as secondary prevention of stroke [9]. Current therapeutic strategies for cognitive impairment include regulation of the cholinergic system via inhibition of acetylcholinesterase (AChE) or direct stimulation of muscarinic and nicotinic receptors, neuroprotection via glutamate-induced N-Methyl D-aspartate (NMDA) receptor overstimulation, and the use of anti-inflammatory and anti-oxidant agents [10–12]. However, cholinesterase inhibitors have been linked to a variety of adverse effects, including gastrointestinal discomfort and bradycardia, among others [13]. Therefore, there is an urgent need to investigate the most effective methods for preventing vascular injury and develop effective and safe treatment options.

People's desire for traditional Chinese medicine for the treatment of VaD has increased in recent years. Naoxintong capsule (NXT), a standardized product of 16 natural components, including 13 plant drugs and 3 animal drugs, namely Radix Astragali seu Hedysari, Radix Angelicae Sinensis, Radix Paeoniae Rubra, Chuanxiong Rhizoma, Carthami Flos, Persicae Semen, Salviae miltiorrhizae radix et rhizome, Achyranthis bidentatae, Spatholobi Stem, Cinnamomi Ranulus, Mori Ramulus, Myrrha, Olibanum, Scorpio, Lumbricus, and Hirudo, has been extensively used in China to treat VaD [14]. The specific characteristics of these 16 natural materials are summarized in Table 1. NXT has been reported to have neuroprotective effects. NXT improves anti-oxidant capacity and prevents calcium overload and reactive oxygen species (ROS) generation, thereby maintaining the mitochondrial membrane potential [15]. NXT protects primary neurons against oxygen-glucose deprivation and reoxygenation (OGD/R) induced injury by inhibiting the mitochondrial apoptotic pathway, which is mediated in part by PI3K-Akt signaling pathway activation [16]. In a previous study, NXT was found to significantly improve the spatial learning-memory ability of VaD mice with chronic hypoperfusion, improve nervous tissue morphology, and inhibit the number of activated astrocytes all at the same time [17]. Other studies have revealed that NXT may reduce the damage of CA1 neurons in rats with ischemic injury and decrease the resting state of hippocampal neurons in vascular dementia model animals [18].

A growing body of research suggests that NXT may improve the memory function and daily behavior ability of VaD patients. Clinical comparative data on treatment regimens and assessment methods, on the other hand, are few. We performed a systematic review and meta-analysis to assess the safety and efficacy of NXT in the treatment of VaD. This study provides fresh insight into future NXT clinical research.

## 2. Materials and Methods

This study was registered with PROSPERO (https://clinicaltrials.gov/ct2/show/CRD42021233199) and carried out in accordance with the PRISMA (Preferred Reporting Items for Systematic Reviews and Meta-analyses) guidelines [19].

### 2.1. Inclusion Criteria

We included all randomized controlled trials (RCTs) that utilized NXT to treat VaD, independent of demographic characteristics, the language of publication, or publication status. While there was no need for allocation concealment or blinding, the included studies had to randomly assign participants to comparison groups. Regardless of gender or age, all participants had VaD with comparable baseline characteristics. The *Diagnostic and Statistical Manual of Mental Disorders* (DSM) or other internationally recognized diagnostic criteria were used to make the VaD diagnosis. The experimental group received NXT alone or in combination with Western medicine (WM) such as AChE inhibitors (donepezil), anti-dementia drugs (memantine), psychostimulants and nootropics (piracetam amd oxiracetam), peripheral vasodilators (duxil, hydergine, buflomedil, and nicergoline), or selective calcium channel blockers with primarily vascular effects (nimodipine and flunarizine). To manage cerebrovascular risk factors or other basic diseases, all patients may get routine treatment (RT), such as anti-hypertensive drugs, anti-diabetics, lipid-lowering drugs, or anti-platelets. At least one of the following outcome indicators was used: mini-mental state examination (MMSE), Montreal Cognitive Assessment (MoCA), Hasegawa dementia scale (HDS), activities of daily living (ADL), or total effective rate (TER).

### 2.2. Exclusion Criteria

We excluded studies that used other Chinese medicine therapies such as Chinese patent medicine, Chinese medicine decoction, and acupuncture, as well as other special therapies such as exercise/physical therapy, psychological intervention, and behavioral interventions. Furthermore, we excluded studies with multiple publications, systematic reviews, case reports, or important data reports, as well as clinical trials where relevant data could not be retrieved or when the corresponding authors could not respond and provide the data.

### 2.3. Outcomes and Definitions

The efficacy evaluation included cognitive functions, the ability of daily living, and the total effective rate. The primary clinical outcome was MMSE. Secondary clinical outcomes included MoCA, HDS, ADL, and TER. MMSE, MoCA, and HDS were used to assess cognitive function, while ADL was used to assess daily living abilities. The TER was mostly determined by the improvement of the aforementioned cognitive function scales. In addition, the occurrence of adverse events (AEs) such as stomach upset, nausea, or loss of appetite was used to assess safety.

### 2.4. Information Sources and Search

Databases such as PubMed, Embase, Web of Science, Cochrane Library, China National Knowledge Infrastructure (CNKI), VIP information resource integration service platform (VIP), and Wanfang Data knowledge service platform (WanFang Data) were searched from inception to September 2021. We included search terms such as “Vascular Dementia,” “Nao Xin Tong,” “Nao Xin Tong,” “Nao XinTong Capsule,” and “Buchang NaoXinTong Capsule,” using methods that combined MeSH terms with free terms.

### 2.5. Study Selection and Data Extraction

Two researchers conducted an independent review of the literature, data extraction, and cross-checking. The third researcher resolved disagreements via discussion or arbitration. To begin, duplicate studies were eliminated using NoteExpress software, and then studies that did not meet the inclusion criteria were eliminated after reading the titles and abstracts. The studies that met the inclusion criteria were thoroughly reviewed, and then data, including general information, methodological information, participant information, interventions, and outcomes, were extracted using Excel software.

### 2.6. Risk of Bias in the Included Studies

Two researchers independently assessed the risk of bias in the included studies using the “risk of bias” evaluation tool in the *Cochrane Handbook for Systematic Reviews of Interventions* (Review Manager, 2014) and relevant assessment guidelines. A total of seven items were included in the risk assessment: (1) random sequence generation, (2) allocation concealment, (3) blinding of participants and personnel, (4) blinding of outcome data, (5) incomplete outcome data, (6) selective reporting, and (7) other bias. According to the evaluation criteria, the seven items were classified as having a “high risk of bias,” “low risk of bias,” or “unclear risk of bias.” The disagreements were resolved by a third researcher via discussion or arbitration.

### 2.7. Data Analysis

Stata 14.0 software was used to conduct the meta-analysis. Continuous variables were analyzed using the weight mean difference (WMD) and 95% confidence interval (CI), while binary variables were analyzed using the odds ratio (OR) and 95% CI. On the other hand, we used the *Q* test and *I*^2^ index to determine the statistical heterogeneity among the included studies [20]. A *P* < 0.05 and *I*^2^ ≥ 50% indicated the presence of statistical heterogeneity. When there was no statistical heterogeneity, the fixed-effects model was used. Otherwise, the random-effects model was used [21]. Both the fixed- and random-effects models used the I-V method. The subgroup analysis was conducted based on clinical heterogeneity. We used funnel plots to conduct a preliminary analysis of publication bias in studies with a sample size greater than or equal to 10. Asymmetry in the distribution of funnel plots suggested a high likelihood of publishing bias. Additionally, Egger's test was used to examine the potential of publication bias. A *P* value greater than 0.05 was shown to be linked with a low likelihood of publication bias. Considering that Western medication encompassed a very heterogeneous category, we conducted a meta-regression analysis to explore its influence on heterogeneity in this study. If necessary, subgroup analysis was conducted according to the type of WM. In order to make the results have more clinical value, the main subgroup analyses were performed according to the treatment approach (NXT vs. blank, NXT + WM vs. WM, and NXT vs. WM). Additionally, to assess the stability and reliability of the study findings, sensitivity analysis was performed by observing the changes in the combined effect and statistical heterogeneity after step-wise elimination of the studies.

### 2.8. Evidence Quality Grade Analysis

The GRADE pro-Guideline Development Tool was used to grade the quality of evidence for the outcomes. There were four levels of evidence quality: high, moderate, low, and very low. RCTs were initially rated as having a high quality of evidence, but it was required to examine if any issues were reducing their quality across five dimensions: risk of bias, inconsistency, indirectness, imprecision, and publication bias, to make a comprehensive judgment [22, 23].

## 3. Results

### 3.1. Search Results

There were 338 publications that met the search strategies from PubMed (*n* = 4), Embase (*n* = 8), the Cochrane Library (*n* = 1), Web of Science (*n* = 11), CNKI (*n* = 106), Wanfang Data (*n* = 112), and VIP (*n* = 96). After screening for duplicates using NoteExpress, a professional document management software, a total of 139 articles were retained. Following a review of the titles and abstracts, 71 articles were excluded, while 35 articles were excluded after a full-text review. Finally, 33 articles were included in the meta-analysis (Figure 1).

### 3.2. Study Characteristics

This study included 33 randomized controlled trials with 2,947 VaD patients (1,486 in the experimental group and 1,461 in the control group) [24–56]. The intervention comparison between the experimental groups and control groups may be summarized as a comparison of three types of treatment strategies: NXT versus blank, NXT + WM versus WM, or NXT versus WM.  Table 2 shows the characteristics of these 33 RCTs. The NXT of all included studies were from the same manufacturer, with the same ingredients. The dosage of NXT was recommended by the instructions. However, the duration of NXT was different, which includes 2, 3, and 6 months.

### 3.3. Risk of Bias in the Included Studies

The randomized allocation was stated in all the 33 studies, whereas 11 studies described the specific allocation methods [24, 26, 30, 32–34, 41, 46, 48, 53, 56]. However, in 3 studies, the random sequence generation was not standardized [32, 46, 48]. None of the studies addressed allocation concealment, and only 1 study used a double-blind method [32]. The remaining 32 studies did not use participant or staff blinding. Furthermore, it was unclear if they used blinding of the outcome data. One study included an outcome indicator: Efficacy Index. However, there was no report for Efficacy Index in the results section, which indicated that it adopted selective reports. Therefore, we evaluated that it had a high risk of reporting bias [50]. However, this had no effect on our analysis (Figures 2 and 3).

### 3.4. Results of the Meta-Analysis

#### 3.4.1. Mini-Mental State Examination (MMSE)

Thirty studies with a total of 2,712 patients showed that the use of NXT in the treatment of VaD improved the MMSE. We used a random-effects model after the heterogeneity test (*I*^2^ = 90.5%, *P* ≤ 0.001). The meta-analysis revealed a significant difference between the experimental group and control group in increasing the MMSE score (WMD = 3.33, 95% CI (2.72, 3.94); Figure 4). A funnel plot analysis of the 30 asymmetrically distributed studies, on the other hand, indicated possible publication bias (Figure 5). Similarly, Egger's test results showed a high likelihood of publication bias (*P*=0.016). Meta-regression analysis showed that the WM category had no significant influence on heterogeneity among studies (*P*=0.082).

*Subgroup Analysis of MMSE*. Subgroup analysis of the MMSE was conducted depending on the treatment approach (NXT vs. blank, NXT + WM vs. WM, and NXT vs. WM; Table 3). The meta-analysis found a significant difference in MMSE between the experimental and control groups in the NXT versus blank subgroup (WMD = 2.99, 95% CI (2.37, 3.94)). Similarly, the results demonstrated a significant difference in MMSE increase between the experimental and control groups in the NXT + WM versus WM subgroup (WMD = 4.15, 95% CI (3.55, 4.75)). In addition, the meta-analysis showed a significant difference in MMSE increase between the experimental and control groups in the NXT versus WM subgroup (WMD = 2.56, 95% CI (1.48, 3.64)).

#### 3.4.2. Montreal Cognitive Assessment (MoCA)

Four studies with a total of 416 patients reported that the use of NXT in the treatment of VaD enhanced the MoCA effect. We used a random-effects model after the heterogeneity test (*I*^2^ = 79.7%, *P*=0.002). The meta-analysis showed that there was a significant difference in increasing the MoCA score between the experimental group and control group (WMD = 4.31, 95% CI (2.72, 5.90); Figure 6). Egger's test results showed that there was little possibility of publication bias (*P*=0.345). Meta-regression analysis showed that the WM category had no significant influence on heterogeneity among studies (*P*=0.096).

*Subgroup Analysis of the MoCA*. Subgroup analysis of the MoCA was performed depending on the treatment approach (NXT vs. blank and NXT + WM vs. WM; Table 3). The meta-analysis found a significant difference in the MoCA increase between the experimental and control groups in the NXT versus blank subgroup (WMD = 2.98, 95% CI (2.21, 3.75)). The meta-analysis results, on the other hand, revealed a significant difference in the MoCA increase between the experimental and control groups in the NXT + WM versus WM subgroup (WMD = 5.61, 95% CI (4.50, 6.73)).

#### 3.4.3. Hasegawa Dementia Scale (HDS)

NXT enhanced the HDS effect in the treatment of VaD, in 9 studies with a total of 917 patients. We used a random-effects model after conducting a heterogeneity test (*I*^2^ = 93.5%, *P* ≤ 0.001). The meta-analysis revealed a significant difference in increasing the HDS score between the experimental group and control group (WMD = 2.71, 95% CI (1.26, 4.17); Figure 7). Egger's test indicated that publication bias was unlikely (*P*=0.058). Meta-regression analysis showed that the WM category was one of the sources of heterogeneity among studies (*P*=0.024).

*Subgroup Analysis of the HDS*. Subgroup analysis of the HDS was performed according to the treatment approach (NXT + WM vs. WM and NXT vs. WM; Table 3). The meta-analysis indicated a significant difference in the HDS increase between the experimental and the control groups in the NXT + WM versus WM subgroup (WMD = 1.26, 95% CI (0.07, 2.45)). The meta-analysis showed a significant difference in the HDS increase between the experimental and control groups in the NXT versus WM subgroup (WMD = 2.90, 95% CI (1.26, 4.55)). Based on the results of meta-regression analysis, the necessary subgroup analysis of the HDS was performed according to the WM category. The meta-analysis indicated a significant difference in the HDS increase between the experimental and the control groups in the nimodipine subgroup (WMD = 0.67, 95% CI (0.25, 1.09), *I*^2^ = 0%) and the Duxil subgroup (WMD = 5.52, 95% CI (4.73, 6.30), *I*^2^ = 12%). In addition, there was only one study report on aniracetam, hydergine, and pyrithioxin dihydrochloride, which could not be pooled because of too few studies.

#### 3.4.4. Activities of Daily Living (ADL)

Fifteen studies with a total of 1,487 patients reported an improvement in ADL when NXT was used to treat VaD. After performing a heterogeneity test (*I*^2^ = 87.6%, *P* ≤ 0.001), we used a random-effects model. The meta-analysis showed a significant difference in ADL score decrease between the experimental group and control group (WMD = −5.85, 95% CI (−7.03, −4.66); Figure 8). On the other hand, a funnel plot analysis of the 15 studies revealed minimal evidence of publication bias due to their very symmetrical distribution (Figure 9). Similarly, Egger's test indicated that publication bias was unlikely (*P*=0.327). Meta-regression analysis showed that the WM category had no significant influence on heterogeneity among studies (*P*=0.790).

*Subgroup Analysis of ADL*. Subgroup analysis of the ADL was conducted based on the different treatment strategies (NXT vs. blank, NXT + WM vs. WM, and NXT vs. WM; Table 3). The meta-analysis revealed a significant difference in the ADL decrease between the experimental and control groups in the NXT versus blank subgroup (WMD = −9.10, 95% CI (−11.33, −6.87)). Similarly, the meta-analysis revealed a significant difference in ADL decrease between the experimental and control groups in the NXT + WM versus WM subgroup (WMD = −5.15, 95% CI (−7.06, −3.24)). In addition, the meta-analysis revealed a significant difference in ADL decrease between the experimental and control groups in the NXT versus WM subgroup (WMD = −5.99, 95% CI (−7.72, −4.26)).

#### 3.4.5. Total Effective Rate (TER)

The TER of NXT in the treatment of VaD was reported in 24 studies with a total of 2,228 patients. The calculation of TER in one study [51] was based on the improvement of MoCA, and 2 studies [33, 56] were based on the improvement of HDS, and the others were based on the improvement of MMSE. We used a fixed-effects model after the heterogeneity test (*I*^2^ = 0.0%, *P*=0.815). The meta-analysis revealed a significant difference between the experimental group and the control group in enhancing the TER (OR = 2.62, 95% CI (2.09, 3.29); Figure 10). A funnel plot analysis of the 24 studies asymmetrically distributed studies indicated the possibility of publication bias (Figure 11); a finding confirmed by the Egger's test (*P* < 0.001). Meta-regression analysis showed that the WM category had no significant influence on heterogeneity among studies (*P*=0.604).

*Subgroup Analysis of TER*. Subgroup analysis of the TER was conducted based on the different treatment strategies (NXT + WM vs. WM and NXT vs. WM; Table 3). The meta-analysis of the NXT + WM versus WM subgroup revealed a significant difference in the TER increase between the experimental and control groups (OR = 3.13, 95% CI (2.29, 4.28)). Additionally, the meta-analysis found a significant difference in the TER increase between the experimental and control groups in the NXT versus WM subgroup (OR = 2.16, 95% CI (1.56, 3.00)).

#### 3.4.6. Adverse Events (AEs)

Twelve studies with a total of 1,247 patients reported AEs associated with the use of NXT to treat VaD. Five studies reported no AEs in either the experimental or control groups. Seven studies reported a total of 29 patients who experienced AEs. The incidence of AEs was 4.65% (29/624). Among them, 28 patients experienced gastrointestinal irritation, whereas only 1 patient reported dizziness. We used a fixed-effects model after the heterogeneity test (*I*^2^ = 0.0%, *P*=0.818). The meta-analysis showed no difference in the occurrence of AEs between the experimental group and control group (OR = 0.72, 95% CI (0.43, 1.22); Figure 12). Additionally, Egger's test showed that publication bias was unlikely (*P*=0.254).

### 3.5. Stratified Analyses

Considering the different duration of NXT among the included studies, we conducted a stratified analysis (Table 4). The meta-analysis revealed that there was no significant difference in increasing the HDS score in the 3-month duration between the experimental group and control group (WMD = 2.18, 95% CI (−0.78, 5.14)). Apart from this, there were significant differences in MMSE, MoCA, HDS, ADL, and TER between the experimental group and the control group in different durations (2, 3, and 6 months). In the NXT versus WM subgroup, there was no significant difference in increasing the HDS score (WMD = 2.18, 95% CI (−0.78, 5.14)) and TER (OR = 1.81, 95% CI (0.87, 3.76)) in the 3-month duration. In the NXT + WM versus WM subgroup, there was no significant difference in decreasing ADL score in the 6-month duration (WMD = −4.07, 95% CI (−12.78, 4.64)). These changes were thought to result from the decrease in sample size.

### 3.6. Sensitivity Analysis

Sensitivity analyses were performed on the MMSE, MoCA, HDS, ADL, TER, and AEs. We serially eliminated one study and performed a meta-analysis of the remaining studies to ascertain changes in the combined effect. The findings indicated that the estimated points were within 95% CI of the total effect, and no directional changes occurred (Figures 13(a)–13(f)). Sensitivity analysis revealed very few changes in the combined effect of the MMSE, MoCA, HDS, ADL, TER, and AEs, thus validating the study findings.

### 3.7. Evidence Quality Grade Analysis

GRADE pro-Guideline Development Tool was used to assess the evidence quality of the following outcomes: MMSE, MoCA, HDS, ADL, TER, and AEs.  Table 5 summarizes the GRADE evidence for outcome measures. The evidence quality of this study was downgraded mainly because of the high risk of bias in the included studies. In addition, the high statistical heterogeneity and publication bias possibility of several outcomes also affect the quality of evidence evaluation. In summary, the evidence quality rating was low.

## 4. Discussion

The purpose of this study was to determine the efficacy and safety of NXT in patients with VaD. The meta-analysis included 33 RCTs with a total of 2,947 patients with VaD. The data indicated that NXT could significantly improve cognitive function and the daily living ability of patients with VaD. NXT was shown to improve the total effective rate of patients without increasing the occurrence of AEs. The most common adverse events associated with NXT were gastrointestinal symptoms, such as stomach upset, nausea, or loss of appetite. Subgroup analysis revealed that whether NXT was used alone or in combination with western medicine, it had the potential to enhance the overall therapeutic effect.

With the increase in the average life expectancy of contemporary individuals, dementia has become a serious public health concern. Worldwide, over 36 million people suffer from dementia, with VaD accounting for at least 20% of all cases [57]. Additionally, the burden of VaD on patients' families, medical care, and long-term care has increased. In many countries, the costs of VaD management have surpassed the cost of cancer or heart disease management. Patients, particularly those who have had a stroke, are at a higher risk of acquiring dementia. Acute stroke was linked with a rapid decrease in cognitive ability that persisted over time in a large population-based study [58, 59]. Therefore, it is important to explore different therapy options that may help VaD patients enhance their cognitive ability and quality of life.

Cholinesterase inhibitors and memantine are the most widely studied drugs for Alzheimer's disease (AD). While the drugs are effective in the treatment of AD, their efficacy in treating VaD is limited. The majority of studies have shown that cholinesterase inhibitors may slightly enhance cognition in patients with VaD (an improvement on the VADAS-cog scale was about 2 points, which was about half of the improvement seen in the AD study). Besides, it has been shown that the cholinesterase inhibitors and memantine improve the overall function of patients with VaD, although evidence on the activities of daily living and behavior remains inconsistent [60]. Previous studies using galantamine in a group of patients with simple VaD and mixed dementia suggested that it may have some advantages. However, many major randomized controlled 6-month trials with galantamine, donepezil, and rivastigmine have been performed with NINDS-AIREN or VaD and reported mixed results [61–63]. On the other hand, although studies on nimodipine in the treatment of subcortical VaD lack key efficacy indicators, they have demonstrated improvements in certain outcomes including memory. In general, there is a dearth of evidence on VaD treatment methods [64]. There is a need to determine the most effective preventive approach and to develop multitargeted therapy alternatives.

Our systematic review indicated that using NXT as monotherapy or adjuvant for VaD patients may be helpful and usually safe. NXT originated from the classic Chinese medicine prescription, “Buyang Huanwu Decoction,” was approved by the China Food and Drug Administration (CFDA) and accepted by the 2015 edition of the Chinese Pharmacopoeia as modern Chinese medicine. NXT was used to invigorate Qi and promote blood circulation. NXT has been used to treat cardiovascular and cerebrovascular diseases such as stroke, coronary heart disease, and angina pectoris for decades. NXT contains 16 Chinese herbal medicines, and more than 200 bioactive constituents have been identified [65]. An HPLC-DAD fingerprint for NXT has been established to represent the character of NXT and to enhance its specificity for quality control and assessment [66]. Previously published research indicated that the traditional Chinese medicine “Buyang Huanwu Decoction” may protect hippocampal cells in the CA1 region [67]. Additionally, prior research has shown that NXT protects against a range of cardiovascular diseases, including atherosclerosis, ischemic stroke, and ischemia-reperfusion injury [65]. NXT ameliorates lipid metabolism and attenuates oxidative inflammation, thus protecting against atherosclerosis. In addition, NXT suppresses ischemia/reperfusion injury-induced activation of the NOD-like receptor pyridine domain-containing protein 3 (NLRP3) inflammasome and IL-1*β* expression [68]. On the other hand, NXT has been demonstrated to recruit and mobilize early endothelial progenitor cells (EPCs)/circulating angiogenic cells (CACs), thereby enhancing the formation of new blood vessels through the VEGF/eNOS signaling [69]. NXT also decreased blood serum levels of Livin, IL-18, and IFN-*γ* contents, and increased VEGF in patients with VaD, thus inhibiting apoptosis and vascular damage. VaD's etiology is very complicated and involves many factors, including lipid metabolism disorder, increased blood viscosity, oxidative damage, or vascular inflammatory stimulation [70]. Indeed, NXT upregulated VEGF expression in ischemic endothelial cells, inhibited endothelial cell apoptosis, and maintained endothelial cell integrity. One of NXT's brain-protective mechanisms has been linked to a decrease in endothelial dysfunction, which promotes angiogenesis and protects ischemic injured nerves.

To assess the effect of NXT on cognitive function, we used the MMSE as the primary outcome indicator coupled with the MOCA or HDS scale. MMSE, MoCA, and NCSE are the most commonly used evaluation methods in previous research [71–74]. We demonstrated that NXT may not only improve cognitive function in VaD patients but also improve overall activities of daily living as measured by the ADL. The evaluation of clinical efficacy is multifaceted. It involves a thorough evaluation of general clinical changes via activities of daily life (functional endpoints) in addition to measuring cognitive function using objective screening tests (cognitive endpoints). Due to the absence of apparent symptoms in patients with mild to moderate VaD, it is difficult to assess symptom improvement. In this case, cognitive ability and overall living ability are used as the primary assessment indicators. Stabilization or improvement of ADL may be a more important endpoint in the late stage of VaD owing to cognitive impairment associated with severe dysfunction. In severe dementia, when cognitive function is unlikely to improve, domain-specific and global as common primary endpoints may be more suitable. In this study, we demonstrated that NXT may also improve daily living activities in patients with VaD, indicating that NXT has multiple protective effects against VaD.

### 4.1. Limitations

The following limitations of this study should be noted. First, the methodological quality of the included studies was generally low. Although all studies explicitly mentioned randomization, only a few studies detailed the method of random grouping. Moreover, none of the studies stated whether or not they used allocation concealment. Only one study used a double-blind design; participants and researchers were not blinded in the other studies. The studies did not specify whether the findings were evaluated blindly. As a consequence, the reliability of the results may be limited. Second, since NXT is a Chinese patent medication, all studies included in this review were conducted in China, and the published articles were written in Chinese, which may lead to potential selection bias. Third, there is no consensus on the most preferred Western medicine for treating VaD, and therefore, a variety of western medicines were used in control groups throughout the included studies. This made it difficult to carry out subgroup analysis according to the types of western medicines. Fourth, MMSE and TER were likely to exhibit publication bias as a consequence of the potential of unreported negative findings, which may decrease the stability of results. For studies with no statistical significance, researchers may consider them of little significance and not publish them or delay publication [75]. Therefore, the improvements in MMSE and TER in this meta-analysis may overestimate the efficacy of the intervention. Fifth, since only four studies with small samples reported MoCA, the findings may be less stable. Sixth, based on the above factors, the current evidence quality of this study was low, so the application in the clinic should be cautious.

## 5. Conclusion

Taken together, our meta-analysis demonstrated that NXT has the potential to enhance the cognitive function and daily living ability of patients without increasing the risk of adverse events whether used alone or in combination with western medicine. This seemed to remind us that NXT may be an effective and safe treatment option for VaD. However, given the low methodological quality of the included RCTs and the quality of current evidence, the findings need to be validated using large sample size, high-quality multicenter RCTs.

## Figures and Tables

**Figure 1:** Flow chart for literature screening.

**Figure 2:** Risk of bias summary.

**Figure 3:** Risk of bias.

**Figure 4:** Forest plot for MMSE of NXT in vascular dementia.

**Figure 5:** Funnel plot for MMSE of NXT in vascular dementia.

**Figure 6:** Forest plot for MoCA of NXT in vascular dementia.

**Figure 7:** Forest plot for HDS of NXT in vascular dementia.

**Figure 8:** Forest plot for ADL of NXT in vascular dementia.

**Figure 9:** Funnel plot for ADL of NXT in vascular dementia.

**Figure 10:** Forest plot for TER of NXT in vascular dementia.

**Figure 11:** Funnel plot for TER of NXT in vascular dementia.

**Figure 12:** Forest plot for AEs of NXT in vascular dementia.

**Figure 13:** Sensitivity analysis: (a) MMSE, (b) MoCA, (c) HDS, (d) ADL, (e) TER, and (f) AEs.

**Table 1:** Details of the NXT.

Chinese name	Pharmaceutical name	Species	Family
Huangqi^∗^	Radix Astragali seu Hedysari	*Astragalus mongholicus Bunge*	Fabaceae
Danggui wei^∗^	Radix Angelicae Sinensis	*Angelica sinensis (Oliv.) Diels*	Apiaceae
Chishao^∗^	Radix Paeoniae Rubra	*Paeonia obovata Maxim*	Paeoniaceae
Chuanxiong^∗^	Chuanxiong Rhizoma	*Ligusticum striatum DC*	Apiaceae
Honghua^∗^	Carthami Flos	*Carthamus tinctorius L*	Asteraceae
Taoren^∗^	Persicae Semen	*Amygdalus sect. Persicae*	Rosaceae
Danshen^∗^	Salviae miltiorrhizae radix et rhizome	*Salvia miltiorrhiza Bunge*	Lamiaceae
Niuxi^∗^	Achyranthis bidentatae	*Achyranthes bidentata Blume*	Amaranthaceae
Jixueteng^∗^	Spatholobi Stem	*Spatholobus suberectus Dunn*	Leguminosae
Guizhi^∗^	Cinnamomi Ranulus	*Cinnamomum cassia (L.) J.Presl*	Lauraceae
Sangzhi^∗^	Mori Ramulus	*Morus alba L.*	Moraceae
Moyao^∗^	Myrrha	*Commiphora myrrha (Nees) Engl*	Burseraceae
Ruxiang^△^	Olibanum	*Boswellia Roxb*	Burseraceae
Quanxie^△^	Scorpio	*Buthus martensii Karsch*	Buthidae
Dilong^△^	Lumbricus	*Pheretima asiatica Michaelsen*	Megascolecidae
Shuizhi^△^	Hirudo	*Leech*	Hirudinidae

^∗^Plant drugs and ^△^animal drugs.

**Table 2:** The baseline characteristics of included studies.

Author	Year	Size (M/F)		Age (year)		Course of disease (month)		Interventions		Duration	Outcomes	AEs (T/C)
		T	C	T	C	T	C	T	C			
Fenghui	2008	22/14	19/13	65.5 ± 14.2	63.9 ± 15.4	6∼28	7∼26	NXT 2# tid + CON-WM	WM: buflomedil hydrochloride	2 m	TER	NA
Gaoli	2012	28/17	27/18	63.8 ± 6.2	65.1 ± 5.6	28.8 ± 14.4	31.2 ± 13.2	NXT 4# tid + CON-WM	WM: nimodipine	3 m (12 w)	MMSE, ADL, TER	NA
Guoqingjun	2013	24/15	21/18	66.9 ± 8.9	64.2 ± 10.0	47.64 ± 11.40	49.44 ± 10.80	NXT 2∼4# tid	WM: nimodipine	6 m	MMSE, HDS, ADL, TER	2/5
Guoweiling	2009	14/16	15/15	65.5 ± 8.53	67.83 ± 8.8	29.16 ± 17.88	34.8 ± 26.76	NXT 3# tid + CON-WM	WM: duxil	6 m	MMSE, TER	NA
Hanxingguo	2007	18/12	17/13	69.4 ± 7.2	68.3 ± 6.6	12	12	NXT 1# tid	WM: hydergine	3 m	MMSE, HDS, TER	None
Huangchaoyun	2004	50	47	64.2 ± 4.8		Unclear		NXT 2# tid	WM: hydergine	2 m (60 d)	TER	NA
Huangdan	2019	25/22	26/21	63.65 ± 2.24	63.21 ± 2.19	Unclear		NXT 4# tid + CON-WM	WM: donepezil	3 m	MMSE, MoCA, TER	3/4
Huanggenxian	2013	21/11	21/11	76.4 ± 7.8	74.0 ± 5.8	35.78 ± 73.20	37.8 ± 67.20	NXT 3# tid	WM: donepezil	2 m (8 w)	MMSE, ADL, TER	None
Huangying	2015	20/16	17/19	70.33 ± 7.47	69.3 ± 7.86	31.59 ± 14.77	31.92 ± 13.85	NXT	WM: flunarizine	6 m	MMSE, ADL	NA
Jiangyouyi	2006	18/12	17/13	65.6 ± 4.2	64.7 ± 5	17.40 ± 15.60	16.68 ± 15.72	NXT 3# tid	WM: duxil	2 m	HDS, TER	NA
Jiangyuan	2014	21/13	19/13	60.38 ± 2.54	60.56 ± 2.34	2.51 ± 3.33	2.62 ± 0.35	NXT 3# tid + CON-WM	WM: donepezil	2 m (8 w)	MMSE, TER	NA
Jinaiguo	2011	35/25	33/27	72.5	71.3	10∼180	7∼190	NXT 3# tid + CON-WM	WM: pyrithioxin dihydrochloride	6 m	MMSE, HDS, ADL, TER	3/4
Lijinyan	2008	47/21	40/26	66.4	62.7	Unclear		NXT 3# tid + CON-WM	WM: hydergine	3 m (90 d)	MMSE, TER	NA
Liwei	2017	23/22	25/20	65.7 ± 6.4	65.6 ± 6.9	Unclear		NXT 4# tid	No WM	6 m	MMSE, MoCA, ADL	NA
Liyanhong	2017	68/51	72/47	66.85 ± 3.96	67.32 ± 7.43	45.96 ± 12.48	50.64 ± 11.76	NXT 3# tid	WM: nimodipine	6 m	MMSE, HDS, ADL, TER	6/8
Liuqingjian	2012	24/17	25/16	61.5 ± 4.3	62.3 ± 5.2	18.0 ± 12.0	20.4 ± 10.8	NXT 4# tid + CON-WM	WM: nimodipine	3 m (12 w)	MMSE, ADL, TER	NA
Liuruixia	2012	16/14	17/13	65 ± 5.1	66.34 ± 6.2	Unclear		NXT 3# tid	WM: piracetam	3 m	MMSE	NA
Manbin	2019	47	47	60.48 ± 6.73	60.61 ± 6.85	34.68 ± 8.88	34.92 ± 9	NXT 3# tid + CON-WM	WM: memantine	2 m	MMSE, MoCA, TER	None
Miaohui	2018	45/24	43/26	68.38 ± 4.57	67.90 ± 6.01	Unclear		NXT 3# tid	No WM	6 m	MMSE, MoCA, AEs	3/0
Shengchenxia	2009	28/17	26/19	66.25 ± 7.16	68.13 ± 8.16	25.68 ± 5.64	26.04 ± 10.92	NXT 3# tid	WM: duxil	3 m (12 w)	MMSE, HDS, ADL, TER	None
Songzhi	2014	25/21	26/20	68.14 ± 4.35	68.17 ± 4.39	28.2 ± 8.04	28.08 ± 8.28	NXT 3# tid	WM: duxil	6 m	MMSE, HDS, ADL	NA
Wangweijia	2011	15/15	15/7	69.9 ± 11.2	66.5 ± 11.2	49.2 ± 22.8	34.8 ± 40.8	NXT 4# tid	WM: duxil	2 m(60 d)	MMSE, TER	NA
Yanfuling	2012	12/17	15/15	70.69 ± 6.98	68.93 ± 8.43	Unclear		NXT 3# tid	WM: nimodipine	3 m(12 w)	MMSE, HDS	NA
Yangping	2019	20/22	21/19	66.3 ± 2.5	65.7 ± 2.6	42.0 ± 9.6	44.4 ± 7.2	NXT 4# tid + CON-WM	WM: nimodipine	3 m	MMSE, TER	NA
Yangxiaoyan	2014	37/13	37/13	65.82 ± 3.19	65.65 ± 3.42	22.32 ± 3.96	24.96 ± 3.72	NXT 4# tid + CON-WM	WM: nimodipine	3 m (12 w)	MMSE, ADL, TER	NA
Yaoxinsheng	2011	22/18	17/19	65.4 ± 6.3	66.2 ± 7.9	21.6 ± 7.2	21.6 ± 9.6	NXT 4# tid + CON-WM	WM: nimodipine	3 m	MMSE, ADL, TER	NA
Yudehai	2012	17/13	15/15	55∼73	56∼75	Unclear		NXT 4# tid	WM: flunarizine	6 m	MMSE, ADL	NA
Yuanlibo	2018	27/20	26/21	67.51 ± 5.67	67.23 ± 5.13	Unclear		NXT 4# tid + CON-WM	WM: oxiracetam + nicergoline	3 m	MMSE, TER	NA
Zhengdejun	2009	30	30	67.8 ± 5.7		Unclear		NXT 2# tid	WM: nimodipine	3 m	MMSE, TER	NA
Zhengtaolin	2014	20/22	22/21	66 ± 7	66 ± 7	Unclear		NXT 3# tid	WM: oxiracetam	3 m(12 w)	MMSE, ADL	None
Zhoulongshou	2013	18/16	19/13	64.3 ± 6.7	57.6 ± 7.8	15.9 ± 9.1	14.8 ± 7.2	NXT 3# tid + CON-WM	WM: donepezil	2 m (8 w)	MMSE, TER, AEs	3/4
Zhouwei	2009	30/30	30/30	70.26 ± 5.21	71.50 ± 5.90	17.30 ± 2.45	18.30 ± 3.22	NXT 4# tid	WM: aniracetam	6 m	MMSE, HDS	9/12
Zhuyingjun	2015	26/29	34/31	55∼84	56∼82	Unclear		NXT 4# tid + CON-WM	WM: nimodipine	6 m	MMSE, ADL, TER	NA

*Note.* T: treatment group, C: control group, M: male, F: female, NXT: Naoxingtong, WM: western medicine, CON-WM: Western medicine of the control group, MMSE: Mini-mental state examination, MoCA: Montreal cognitive assessment, HDS: Hasegawa dementia mcale, ADL: activities of daily living, TER: total effective rate, AEs: adverse events, d: day, w: week, m: month, and NA: not mentioned.

**Table 3:** Results of the subgroup analysis based on different treatment strategies.

	Subgroup	Studies	Participants	WMD (95% CI)/OR (95% CI)	*I* ^2^	*P*
MMSE	Overall	30	2,712	3.33 (2.72, 3.94)	90.5%	＜0.001
	NXT vs. blank	2	228	2.99 (2.37, 3.61)	0.0%	0.903
	NXT + WM vs. WM	14	1,301	4.15 (3.55, 4.75)	77.4%	＜0.001
	NXT vs WM	14	1,183	2.56 (1.48, 3.64)	90.2%	＜0.001

MoCA	Overall	4	416	4.31 (2.72, 5.90)	79.7%	0.002
	NXT vs. blank	2	228	2.98 (2.21, 3.75)	0.0%	0.897
	NXT + WM vs. WM	2	188	5.61 (4.50, 6.73)	0.0%	0.573
	NXT vs. WM	0	0	—	—	—

HDS	Overall	9	917	2.71 (1.26, 4.17)	93.5%	＜0.001
	NXT vs. blank	0	0	—	—	—
	NXT + WM vs. WM	1	120	1.26 (0.07, 2.45)	—	—
	NXT vs. WM	8	797	2.90 (1.26, 4.55)	94.3%	＜0.001

ADL	Overall	15	1,487	−5.85 (−7.03, −4.66)	87.6%	＜0.001
	NXT vs. blank	1	90	−9.10 (−11.33, −6.87)	—	—
	NXT + WM vs. WM	6	618	−5.15 (−7.06, −3.24)	91.4%	＜0.001
	NXT vs. WM	8	779	−5.99 (−7.72, −4.26)	84.9%	＜0.001

TER	Overall	24	2,228	2.62 (2.09, 3.29)	0.0%	0.815
	NXT vs. blank	0	0	—	—	—
	NXT + WM vs. WM	15	1,369	3.13 (2.29, 4.28)	0.0%	0.714
	NXT vs. WM	9	859	2.16 (1.56, 3.00)	0.0%	0.888

**Table 4:** Results of the stratified analysis based on different NXT duration.

Subgroup		Overall		2-month duration		3-month duration		6-month duration	
		Studies	WMD (95% CI)/OR (95% CI)	Studies	WMD (95% CI)/OR (95% CI)	Studies	WMD (95% CI)/OR (95% CI)	Studies	WMD (95% CI)/OR (95% CI)
MMSE	Overall	30	3.33 (2.72, 3.94)	5	3.37 (2.10, 4.65)	14	3.35 (2.35, 4.34)	11	3.28 (2.17, 4.40)
	NXT vs. blank	2	2.99 (2.37, 3.61)	0	—	0	—	2	2.99 (2.37, 3.61)
	NXT + WM vs. WM	14	4.15 (3.55, 4.75)	3	4.27 (3.27, 5.28)	8	4.66 (4.28, 5.04)	3	2.88 (0.26, 5.50)
	NXT vs. WM	14	2.56 (1.48, 3.64)	2	1.84 (0.81, 2.87)	6	1.73 (0.81, 2.66)	6	3.56 (1.76, 5.36)

MoCA	Overall	4	4.31 (2.72, 5.90)	1	6.02 (4.22, 7.82)	1	5.36 (3.93, 6.79)	2	2.98 (2.21, 3.75)
	NXT vs. blank	2	2.98 (2.21, 3.75)	0	—	0	—	2	2.98 (2.21, 3.75)
	NXT + WM vs. WM	2	5.61 (4.50, 6.73)	1	6.02 (4.22, 7.82)	1	5.36 (3.93, 6.79)	0	—
	NXT vs. WM	0	—	0		0	—	0	—

HDS	Overall	9	2.71 (1.26, 4.17)	1	5.00 (3.60, 6.40)	3	2.18 (-0.78, 5.14)	5	2.59 (0.63, 4.54)
	NXT vs. blank	0	—	0	—	0	—	0	—
	NXT + WM vs. WM	1	1.26 (0.07, 2.45)	0	—	0	—	1	1.26 (0.07, 2.45)
	NXT vs. WM	8	2.90 (1.26, 4.55)	1	5.00 (3.60, 6.40)	3	2.18 (−0.78, 5.14)	4	2.94 (0.41, 5.47)

ADL	Overall	15	−5.85 (−7.03, −4.66)	1	−4.03 (−7.01, −1.05)	6	−5.82 (−6.95, −4.68)	8	−6.11 (−8.49, −3.73)
	NXT vs. blank	1	−9.10 (−11.33, −6.87)	0	—	0	—	1	−9.10 (−11.33, −6.87)
	NXT + WM vs. WM	6	−5.15 (−7.06, −3.24)	0	—	4	−5.58 (−7.22, −4.48)	2	−4.07 (−12.78, 4.64)
	NXT vs. WM	8	−5.99 (−7.72, −4.26)	1	−4.03 (−7.01, −1.05)	2	−5.69 (−8.09, −3.30)	5	−6.39 (−8.71, −4.06)

TER	Overall	24	2.62 (2.09, 3.29)	8	2.58 (1.66, 4.01)	10	3.31 (2.26, 4.86)	6	2.16 (1.50, 3.09)
	NXT vs. blank	0	—	0	—	0	—	0	—
	NXT + WM vs. WM	15	3.13 (2.29, 4.28)	4	2.73 (1.37, 5.44)	8	4.15 (2.65, 6.49)	3	2.21 (1.27, 3.86)
	NXT vs. WM	9	2.16 (1.56, 3.00)	4	2.48 (1.40, 4.41)	2	1.81 (0.87, 3.76)	3	2.12 (1.32, 3.40)

**Table 5:** GRADE evidence summary of outcome measures.

Outcomes	Certainty assessment							Patients		Effect	Quality
	*N*	Design	Risk of bias	Inconsistency	Indirectness	Imprecision	Others	*T*	*C*	WMD/OR (95% CI)	
MMSE	30	RCTs	Serious^1^	Serious^2^	No serious	No serious	Serious^3^	1,366	1,346	3.33 (2.72, 3.94)	Very low
MoCA	4	RCTs	Serious^1^	Serious^2^	No serious	No serious	No serious	208	208	4.31 (2.72, 5.90)	Low
HDS	9	RCTs	Serious^1^	Serious^2^	No serious	No serious	No serious	458	459	2.71 (1.26, 4.17)	Low
ADL	15	RCTs	Serious^1^	Serious^2^	No serious	No serious	No serious	745	742	−5.85 (−7.03, 4.66)	Low
TER	24	RCTs	Serious^1^	No serious	No serious	No serious	Serious^3^	973/1,128	779/1,100	2.62 (2.09, 3.29)	Low
AEs	12	RCTs	Serious^1^	No serious	No serious	No serious	No serious	29/624	37/623	0.72 (0.43, 1.22)	Moderate

^1^Lack of random method, blinding, and allocation concealment of reporting; ^2^*I*^2^ ≥ 50%; ^3^Suspicion of publication bias; *N*: number of studies; *T*: treatment group; and *C*: control group.

## Data Availability

The data used to support the findings of this study are included within the article.

## Abbreviations

VaD: Vascular dementia
FDA: Food and drug administration
AChE: Acetylcholinesterase
NMDA: N-methyl D-aspartate
NXT: Naoxintong capsule
PRISMA: Preferred reporting items for systematic reviews and meta-analyses
RCTs: Randomized controlled trials
DSM: Diagnostic and statistical manual of mental disorders
WM: Western medicine
RT: Routine treatment
MMSE: Mini-mental state examination
MoCA: Montreal Cognitive Assessment
HDS: Hasegawa dementia scale
ADL: Activities of daily living
TER: Total effective rate
AEs: Adverse events
CNKI: China National Knowledge Infrastructure
WMD: Weight mean difference
CI: Confidence interval
OR: Odds ratio
CFDA: China food and drug administration
NLRP3: Domain-containing protein 3
EPCs: Endothelial progenitor cells
CACs: Circulating angiogenic cells
ROS: Reactive oxygen species
OGD/R: Oxygen-glucose deprivation and reoxygenation.

## Additional Points

(i) Naoxintong capsule has good efficacy on vascular dementia. (ii)·Naoxintong Capsule has good safety for vascular dementia. (iii)·Naoxintong Capsule may be an effective and safe way for vascular dementia.
